# Polyextremotolerant black fungi: oligotrophism, adaptive potential, and a link to lichen symbioses

**DOI:** 10.3389/fmicb.2012.00390

**Published:** 2012-11-08

**Authors:** Cene Gostinčar, Lucia Muggia, Martin Grube

**Affiliations:** ^1^Department of Biology, Biotechnical Faculty, University of LjubljanaLjubljana, Slovenia; ^2^Centre of Excellence for Integrated Approaches in Chemistry and Biology of ProteinsLjubljana, Slovenia; ^3^Institute of Plant Sciences, Karl-Franzens-University GrazGraz, Austria; ^4^Department of Life Science, University of TriesteTrieste, Italy

**Keywords:** melanin, oligotrophism, secondary metabolites, protective molecules, stress

## Abstract

Black meristematic fungi can survive high doses of radiation and are resistant to desiccation. These adaptations help them to colonize harsh oligotrophic habitats, e.g., on the surface and subsurface of rocks. One of their most characteristic stress-resistance mechanisms is the accumulation of melanin in the cell walls. This, production of other protective molecules and a plastic morphology further contribute to ecological flexibility of black fungi. Increased growth rates of some species after exposure to ionizing radiation even suggest yet unknown mechanisms of energy production. Other unusual metabolic strategies may include harvesting UV or visible light or gaining energy by forming facultative lichen-like associations with algae or cyanobacteria. The latter is not entirely surprising, since certain black fungal lineages are phylogenetically related to clades of lichen-forming fungi. Similar to black fungi, lichen-forming fungi are adapted to growth on exposed surfaces with low availability of nutrients. They also efficiently use protective molecules to tolerate frequent periods of extreme stress. Traits shared by both groups of fungi may have been important in facilitating the evolution and radiation of lichen-symbioses.

Most research of fungal biology is centered on relatively fast-growing fungi that can easily be cultured in mesophilic and axenic conditions. This hardly reflects the situation in nature, which is frequently characterized by changing abiotic conditions, resource limitation, and different interactions with other organisms. Those organisms specialized for habitats with low availability of nutrients and symbiotic organisms are often slow-growing and very difficult to study by genetic manipulation; their biology is therefore still poorly understood. Due to increased accessibility of high-throughput methods, such as next-generation sequencing, significant resources are now dedicated to generating and mining large amounts of genomic, transcriptomic, and proteomic data in search of determinants of stress-tolerance, also for many non-model organisms. Although this approach is powerful, it is not exhaustive, as has been demonstrated by a recent breakthrough in studying the radiotolerant bacterium *Deinococcus radiodurans*. Large scale “omics” studies showed only that extreme radiation resistance of this bacterium is not caused by unusually efficient DNA repair mechanisms as initially presumed. The mechanisms of radiotolerance seemed more enigmatic then ever, until a set of elegant non-“omics” experiments showed that the key adaptation is much simpler: it is based on the accumulation of antioxidant manganese orthophosphate and peptide complexes that protect the cell proteome (Daly et al., 2010).

In studying fungal extremotolerance, too, the sometimes noticed perception of the omnipotence of “omics” should be avoided. Instead, more focus should be given to other approaches, with the aim of investigating alternative levels of adaptation to extreme stress. Two of them will be presented here: (1) accumulation of melanin and other metabolites with different protective roles, (2) growth in oligotrophic conditions by interaction with other microorganisms or by employing unusual metabolic pathways.

## Melanin as a versatile polymer of oligotrophic fungi

Many oligotrophic fungi respond to stress conditions by expressing a high degree of phenotypic plasticity (Slepecky and Starmer, 2009; Gostinčar et al., 2010). This is particularly well-exemplified by the so-called black fungi (also known as “black yeasts” or “black meristematic fungi”), a polyphyletic group of fungi which share several peculiar phenotypic traits. Depending on the environmental conditions, these fungi can shift between yeast-like, filamentous, and meristematic (isodiametrical, resulting in a small surface/volume ratio) growth. Besides this the most visually prominent adaptation is frequently in the production of melanin—the substance that earned black fungi their name.

Melanin is a protective dark pigment in the cell walls that facilitates the survival of the harsh conditions. Melanins of black fungi are different types of high molecular weight pigments produced by the coupling of phenolic units. Different metabolic sources deliver necessary precursors of fungal melanins, including 3, 4-dihydroxyphenylalanine, γ-glutaminyl-3, 4-dihydroxybenzene, catechol and 1, 8-dihydroxynaphthalene. The coupling of these precursors to complex macromolecules is accomplished enzymatically, but the details are still poorly understood (among the candidate enzymes are extracellular phenoloxidases, laccases, tyrosinases, catalases, and peroxidases; Butler and Day, 1998).

Melanin plays an important role in the ability of melanized fungi to survive excessive heat or cold, extreme pH or osmotic conditions, polychromatic UV-radiation, simulated space and Martian conditions, and it also seems to mediate tolerance toward metals (Gadd and de Rome, 1988; Gunde-Cimerman et al., 2000; Onofri et al., 2008; Sterflinger et al., 2012). Some of melanized species are strikingly tolerant to ionizing radiation and have been found in nuclear reactors and reactor cooling water (Zhdanova et al., 2000). They even seem to be able to use their melanin to convert ionizing gamma radiation into chemical energy by still unknown mechanisms (Dadachova et al., 2007). Metabolic responses of melanin-producing fungi to ionizing radiation include increasing rates of electron transfer, measured as reduction of ferricyanide by the reduced nicotinamide adenine dinucleotide (NADH) (Dadachova et al., 2007). Gamma radiation-induced oxidation of melanin resulted in electric current production, especially in the presence of a reducing agent (Turick et al., 2011). The biological significance of this phenomenon is still unclear and some experiments yield contradicting results: gamma radiation, UV, and visible light seem to cause a reduction of ATP levels in melanized cells of the fungus *Cryptococcus neoformans* (Bryan et al., 2011).

## Protective compounds in black fungi and other stress-tolerant fungi

Beside the versatile polymer melanin, other protective compounds aid in pursuing an oligotrophic and stress-tolerant life style. Among these, mycosporines are efficient absorbers of UV radiation, with the maximum absorbance between 310 and 365 nm. Mycosporines and mycosporine-like amino acids (MAAs) comprise low-molecular-weight (generally less than 400 Da), water-soluble molecules composed of either an aminocyclohexenone or an aminocycloheximine ring, carrying nitrogen, or imino alcohol substituents. When substituted with amino acid residues, they are designated MAAs. They act as shields against UV radiation, but some MAAs may also protect the cell by scavenging reactive oxygen species such as singlet oxygen, superoxide anions, hydroperoxyl radicals, and hydroxyl radicals. Additionally, a function of mycosporines as compatible solutes has been suggested in fungi (Gorbushina et al., 2003; Kogej et al., 2006). These fungi had a significantly higher content of mycosporine glutaminol-glucoside when grown in 10% salt than in a salt-free medium. Besides black yeasts, mycosporines are synthesized by many other fungal species as well as non-fungal microorganisms (reviewed in Oren and Gunde-Cimerman, 2007).

Accumulation of trehalose as a stress protectant has been extensively studied, especially in the example of *Saccharomyces cerevisiae* (Shima and Takagi, 2009), but also in other fungi (Ocon et al., 2007). Additional compounds with similar functions and widespread fungal occurrence include polyalcohols, betaine, and proline (Blomberg and Adler, 1992; Takagi, 2008; Shima and Takagi, 2009). Various carotenoid pigments (e.g., torularhodin or astaxanthin) have been suggested to scavenge the reactive oxygen species in red yeasts and protect them from UV damage (Madhour et al., 2005). Not dissimilar to the role of manganese in the bacterium *D. radiodurans* (Daly et al., 2010) some findings on *S. cerevisiae* indicate the importance of manganese homeostasis in prevention of oxidative damage in the absence of superoxide dismutase (Lapinskas et al., 1995). Although compounds with protective functions are also produced by stress-sensitive organisms, their accumulation is of fundamental importance for persistence and survival in extremotolerant life forms.

Fungi that pursue a self-sustaining symbiotic life-style with algae (lichen symbioses) appear to be especially adept at synthesizing stress protective compounds (Boustie et al., 2011). Among others, protective strategies include physical light scattering mediated by oxalates or UV-absorbers, such as xanthophylls, carotenoids, or more typical lichen compounds, such as dibenzofuranes (e.g., usnic acid), depsides (e.g., atranorin), depsidones (e.g., lobaric acid), or shikimate derivatives (e.g., calycin). In lichens involving fungal-cyanobacterial symbioses, only oxo-carbonyl mycosporines of likely fungal origin were previously found (Rezanka et al., 2004), but recently, several new types of mycosporines were detected in various species (Roullier et al., 2009, 2011). Known secondary compounds also seem to act as antioxidants (Boustie et al., 2011), and discovery of more such compounds is ongoing. Ramalin [γ-glutamyl-N'-(2-hydroxyphenyl)hydrazide] from the Antarctic lichen *Ramalina terebrata* is a novel compound with antioxidant function (Paudel et al., 2011). Most of the lichen compounds accumulate as crystals on the external surfaces of hyphae (as extrolites). They occasionally represent as much as half of 5–20% of material extractable with organic solvents (Boustie et al., 2011).

## Ubiquity of the oligotrophic lifestyle

Ancestors of black fungi from the large lineages of Dothideomycetes and Chaetothyriomycetidae (which evolved much later) were presumably oligotrophic organisms living on rock surface or subsurface (Gueidan et al., 2011). Rocks, as the most abundant natural substrate of oligotrophic black fungi, are colonized in all climatic zones, including the most hostile environments on Earth such as Antarctic dry valleys, the Atacama Desert, or high alpine habitats in the Himalayas (Onofri et al., 2007; Selbmann, pers. comm.). Their radiotolerance could have helped them to survive and proliferate during historic periods of increased cosmic radiation, e.g., due to weakened or absent magnetic field of the Earth (Dadachova and Casadevall, 2008). Similar to the bacterium *D. radiodurans*, radiotolerance in black fungi is tightly linked to pronounced desiccation-tolerance (which may have actually been the primary function of the adaptations; Daly, 2012). Consequently these fungi appear to prevail in habitats with only sporadic availability of water (alternating humidity, rain, and condensation).

Oligotrophic fungi can also grow in anthropogenic habitats; they are very common on monuments, concrete walls, and similar rock-like surfaces where they can cause undesirable coloration (Hallmann et al., 2011; Miller et al., 2012). They are also present on glass, metals, or silicon, and on a wide variety of more or less durable organic surfaces such as plastic materials and other polymers (Gostinčar et al., 2011), which they might help to degrade. At least some oligotrophic fungi can use complex phenolic hydrocarbons from the environment as the sole source of carbon and energy. Such fungi are commonly found in unusual habitats, such as biofilters or distilleries (Prenafeta-Boldu et al., 2006; Scott et al., 2007). Several of these species are closely related to human pathogens, therefore it has even been argued that there is a physiological connection between aromatic hydrocarbon assimilation and capability of mammalian infection (Prenafeta-Boldu et al., 2006).

## Unusual sources of energy and carbon?

In addition to their cohabitation with algae, the ubiquity of black fungi on rocks in polar and other largely unpolluted areas indicates the possible existence of unpredicted and unconventional ways of carbon acquisition or energy gain. In this context, Palmer and Friedman (1988) suggested first evidence for aerial CO_2_ uptake by a black fungus isolated from Antarctic cryptoendolithic communities after ^14^C-labeling experiments. These results, as exciting as they seem, are still pending confirmation by modern approaches. They could explain the occurrence of black fungi in other unusual habitats, e.g., on gypsum (CaSO_4_) surfaces in Atacama Desert (de los Rios, pers. comm.), where they cannot derive substantial amounts of fixed carbon from the substrate.

Besides carbon, energy sources in such environments can be equally scarce. It is tempting to speculate how radiation of different wavelengths could be transformed into biochemical energy. The possible role of melanin has already been mentioned above. Besides that energy production could involve proteins of the plasma membrane. Intriguing candidates for such function are the light-sensing rhodopsins. Bacteriorhodopsin has been first discovered four decades ago in the cell membrane of the archaeon *Halobacterium* sp., where it functions as a light driven proton pump (Grote and O'Malley, 2011). Although numerous homologues of bacteriorhodopsins have been described in fungal genomes since then, little information exists on their (probably versatile) functions (Fan et al., 2011). Some of them may act as photosensors, however, in the case of the black fungus *Leptosphaeria maculans* a bacteriorhodopsin-like proton pump was shown to use the energy of photons to pump protons out of the cell and therefore transform radiation energy into the chemical form—the transmembrane proton gradient (Waschuk et al., 2005). It is not difficult to imagine the possible uses for this electrochemical potential. Proton gradient for example appears to be crucial for the halotolerance of the black fungus *Hortaea werneckii*. It supplies transmembrane transporters with the energy for maintaining the appropriate intracellular concentration of anorganic ions and compatible solutes (Gostinčar et al., 2011).

A further question is whether the atmospheric carbon dioxide could be routed into the fungal metabolism, although it lacks a Calvin cycle comparable to that found in plants. Alternative pathways of carbon fixation are already known from prokaryotes (Fuchs, 2011). It is often overlooked that these prokaryotic pathways contribute to the global carbon cycle and that most likely more pathways still remain to be discovered. Each of the alternative carbon fixation pathways has its own characteristics that are related to the ecology of the organism. They differ in their energy budget and in their sensitivity to oxygen (Bar-Even et al., 2012). Almost surprisingly, no oligotrophic eukaryote has so far been studied for carbon fixation beyond the Calvin cycle. Although such mechanisms might be irrelevant for fungi when they live in nutrient-rich habitats, they could still represent a life-sustaining option for slow-growing oligotrophic rock fungi in competitor-free environments (Parkinson et al., 1989, 1990; and references therein).

## Incipient symbiotic associations and a possible link with the lichen-life style

What other options are available to oligotrophic black fungi growing on surfaces with almost no usable organic-carbon? Some evidence shows that black fungi improve their carbon supply by attaching to microscopic algae (Figure 1). Rock-inhabiting and lichen-inhabiting microcolonial fungi develop into lichenoid structures within months when co-cultured with lichen algae (Gorbushina et al., 2005; Brunauer et al., 2007). Black fungi and lichens often co-occur on the same pieces of rock, and in arid habitats, black fungi are commonly visible as lichen colonizers (Harutyunyan et al., 2008). Recently, Gorbushina and Broughton (2009) interpreted the rock surface as a kind of “symbiotic playground,” where they considered antibiosis (detrimental interactions between species) to be rare and counterproductive. The authors also mentioned—without providing further details—that co-cultivation of the cynobacterium *Nostoc* with a rock-inhabiting fungus (*Sarcinomyces*) resulted in a specific spatial arrangement of both organisms and growth alteration in the photosynthetic cyanobacteria.

**Figure 1:** **When do we call it lichen? (A)** Lichen-like association of *Cladosporium*-like fungus (according to ITS sequences) with aerial algal cells, on polypropylene surface, Botanical Garden Graz, 2011. Arrows indicate coccal algal cells (a) attached to fungal hypha (f); Bar = 20 μm. **(B)** Habit of the “black” lichen *Cystocoleus ebeneus*; a closed sheath of black fungal hyphae (f) wrap a central algal thread (a); Bar = 10 μm.

An ancestral proximity of certain lichenized fungal lineages and different lineages of black fungi has been shown by reconstructing their molecular phylogeny. Rock-inhabitants are basal to the large lichenized lineages of Arthoniomycetes and Verrucariales (Gueidan et al., 2008; Ruibal et al., 2009). In these groups we also find complex morphologies (stratified lichen thalli that also include shrub- or leaf-like habits). The lichen lifestyle is not predominant in Dothideomycetes and is scattered in different clades within this class (Muggia et al., 2008; Nelsen et al., 2009; Figure 2). Also, lichen thallus morphology in Dothideomycetes is generally simple (Figure 1B).

**Figure 2:** **Close relationships of life styles in a subgroup of the *Teratosphaeriaceae* (Dothideomycetes), including rock-inhabiting black fungi and lichens, and plant-surface colonizers.** Bayesian analysis of combined nuSSU, nuLSU, mtSSU, and rRNA genes.

Loose associations of black fungi and algae in nature might be seen as borderline lichens (Kohlmeyer et al., 2004), without development of complex symbiotic textures of the fungi (Figure 1A). We interpret such forms as primitive stages of lichenization and as contemporary analogs of early lichen evolution. It is likely that a transition from the rock-inhabiting to the lichenized lifestyle of fungi in early ascomycetous evolution is connected to their exquisite stress physiology. Desiccation and irradiation increase the formation of reactive oxygen species in both fungi and algae, but the lichen symbiosis increases the efficiency of the protective mechanisms compared to isolated symbiotic partners (Kranner et al., 2005). These mechanisms involve the glutathione redox system, which is also known from black fungi (Jürgensen et al., 2001). In addition, small protective molecules that accumulate in black fungi as stress-responsive osmolytes could be involved in the transition from rock-inhabiting to the lichen life style. Polyols such as ribitol, sorbitol, and erythritol, as well as glucose, provided by algae and cyanobacteria, respectively, are taken up by lichen fungi as food molecules and transformed to mannitol (Friedl and Büdel, 2008). Efficient osmolyte metabolism, as found in oligotrophic black fungi, might serve as a pre-adaptation to facilitate the transition to a lichen symbiotic life style.

Knowledge about stress-protective mechanisms in black fungi and lichenized fungi may lead to unforeseen applications in medicine and industry. This was exemplified recently in the case of protective molecules from the bacterium *D. radiodurans*. These were shown to preserve immunogenicity of epitopes during sterilisation of the pathogen by gamma radiation, opening new possibilities for vaccine development (Gaidamakova et al., 2012). In fungi MAAs can be used as a UV filter and have already been commercialized in suncare products (Rastogi et al., 2010). In a similar manner the radioprotective properties of melanin could be used to shield bone marrow during cancer radiotherapy (Schweitzer et al., 2010). The vast diversity of other compounds from lichens still needs to be screened for potential beneficial properties (Boustie et al., 2011).

As rapid progress in sequencing technologies will enable us to look deeper into the genomes of non-conventional, oligotrophic organisms, analyses of previously unimaginable amounts of data will answer many, but not all, questions about their biology. Besides the presence of stress-associated genes and expressed products, other mechanisms appear to play an important role in the linked phenomena of polyextremotolerance and oligotrophism. These include small metabolites and their complexes. Therefore the bioinformatic rush following the “omics” revolution needs to be accompanied by well-designed, hypothesis-driven experimental work to evaluate phenotypic plasticity, production of multi-purpose protective metabolites, and metabolic interactions with other microorganisms as responses to a life in hostile environments.

## Conflict of interest statement

The authors declare that the research was conducted in the absence of any commercial or financial relationships that could be construed as a potential conflict of interest.
